# Women living with HIV and dual contraceptive use in Ethiopia: systematic review and meta-analysis

**DOI:** 10.1186/s40834-022-00179-8

**Published:** 2022-07-02

**Authors:** Asteray Ayenew

**Affiliations:** Midwifery Department, College of Medicine and Health Sciences, Bahir Dar University, Bahir Dar, Ethiopia

**Keywords:** Dual contraceptive use, Women living with HIV, Systematic review and meta-analysis, Ethiopia

## Abstract

**Background:**

Despite different preventive strategies that have been implemented in the country, the prevalence of HIV/AIDS is still significantly increasing in Ethiopia. The concurrence of HIV and unintended pregnancy makes the use of dual contraception a back bone for the simultaneous protection against HIV, and unintended pregnancy. As a result, this systematic review and meta-analysis aimed to assess the prevalence and associated factors of dual contraceptive use among women living with HIV in Ethiopia.

**Method:**

We used databases; (PubMed, Google Scholar, EMBASE, Cochrane Library, African Online Journals, and Hinary), other gray and online repository accessed studies were searched using different search engines. For critical appraisal of studies Newcastle-Ottawa Quality Assessment Scale (NOS) was used. The analysis was done using STATA 11 software. The Cochran Q test and I^2^ test statistics were used to assess the heterogeneity. To detect publication bias funnel plot and Egger’s test were used. The pooled prevalence of dual contraception use and the odds ratio (OR) with a 95% confidence interval was presented by using forest plots.

**Result:**

Eleven studies were included in this review, with a total of 4083 women living with HIV in Ethiopia. The pooled prevalence of dual contraception use in Ethiopia was 34.08% (95%CI: 20.77–47.38). Having open partner discussion (OR = 3.96, 95%CI:2.3,6.8), provision of post test counseling (AOR = 4.38, 95%CI:2.93,6.54), disclosed HIV status to sexual partners (OR = 5.9, 95%CI:4.19,8.33), partner involvement in post-test counseling (OR = 3.52, 95%CI:2.37,5.23), and being on highly active antiretroviral therapy (HAART) (OR = 2.9, 95%CI:1.56,5.46) were the determinant factors of dual contraceptive use in Ethiopia.

**Conclusion:**

The overall prevalence of dual contraceptive use among women living with HIV in Ethiopia was low. Having open partner discussion, provision of post-test counseling, disclosed HIV status to sexual partner, partner involvement in post-test counseling, and currently on highly active antiretroviral therapy (HAART) were the associated factors of dual contraceptive use. Therefore, efforts should be made to provide post-test counseling, and initiate partner involvement in post-test counseling. Moreover, promoting open partner discussion, counseling to disclose HIV status to their sexual partner and to start HAART will be helpful in enhancing the use of dual contraceptive method use.

## Background

Globally, more than 36.7 million people were living with human immune deficiency virus (HIV) [1]. The problem is highest among people residing in Sub Saharan Africa where, 60% of people reported to live with human immune deficiency virus/acquired immune deficiency syndrome (HIV/AIDS) and more than half of them were females [2]. The total number of people living with HIV in Ethiopia was 769, 600 in 2014. Of these females cover more than 60% [3].

HIV/AIDS continues to have disastrous medical, social, economic, and physical impacts on individuals, nations and the global community at large [4]. Unintended pregnancies accounted for 21.3% of new pediatric HIV infections, and 90% were from Sub Saharan Africa [5, 6]. In Ethiopia, annually, over 100, 000 pregnancies tested positive for HIV and over 12, 000 HIV-positive births. Unintended pregnancies contribute to poor maternal and child outcomes especially among HIV infected women [7, 8].

Dual protection can be achieved through the use of barrier method (condoms) or dual method (condoms + another modern contraceptive method) use [9]. Dual contraception can be an effective strategy to prevent HIV transmission to partners, prevalence of mother to child transmission, and to prevent unintended pregnancy. Evidence show that 40 and 80% of unplanned pregnancies and abortions would be prevented if half and all of them who were using one type of contraceptive alone started using dual methods [10]. Additionally, an interventional based study had also demonstrated that adherence to the dual contraception lower the rate of unintended pregnancy at 24 months [11].

Currently, in Ethiopia, HIV transmission is very high and is a major public health problem. to Due to low dual contraceptive method use, many HIV positive women are still facing unintended pregnancy, and its complication with a concomitant risk of mother to child transmission (MTCT) of HIV, pregnancy related morbidity and mortality. The national health policy of Ethiopia recommends the use of dual contraception as a key intervention to reduce transmission of HIV/AIDS, PMTCT, and unintended pregnancy. Additionally, the Ministry of health in collaboration with partners developed the post 2015 objective of prevention of mother-to-child transmission (PMTCT) to consolidate & sustain the elimination of MTCT and reduce the vertical transmissions to less than 2% by 2020. To ensure virtual elimination, one of the main focuses is improving the use of dual protection among HIV positive women by integrating family planning services with PMTCT [12]. As a result, this systematic review and meta-analysis aimed to estimate the pooled prevalence of dual contraception use among women living with HIV and its associated factors in Ethiopia.

## Methods

This systematic review and meta-analysis were conducted to estimate the national use of dual contraception and its associated factors among women living with HIV in Ethiopia. We used the Preferred Reporting Items for Systematic Reviews and Meta-Analyses (PRISMA) checklist guideline [13].

### Searching strategy

First, the PROSPERO database and database of abstracts of reviews of effects (DARE) (http://www.library.UCSF.edu) were searched to check whether published or ongoing projects exist related to the topic. The literature search strategy, selection of studies, data extraction, and result reporting were done in accordance with the Preferred Reporting Items for Systematic Reviews and Meta-Analyses (PRISMA) guidelines [14]. We searched PubMed, Google Scholar, EMBASE, Cochrane Library, HINARI, WHO Afro Library Databases, and African Online Journal databases for all available studies using the following terms: “dual contraception use” OR “dual protection” OR “condom” AND “sexually active women living with HIV” OR “condom” OR “modern contraception” OR “use of dual methods” OR “prevalence” OR “determinants” AND Ethiopia”. The search string was developed using “AND” and “OR” Boolean operators. Searching terms were based on adapted PICO principles to search through the above-listed databases to access all the relevant articles. For unpublished studies, the official websites of Ethiopian’s University research repository online library (University of Gondar and Addis Ababa University) was used.

### Inclusion and exclusion criteria

Studies reported the prevalence and/or associated factors, or determinant factors of dual contraception method use were included in this study. English language literature and research articles only were included. Whereas articles without full text and abstract, anonymous reports, duplicate studies and editorial reports were excluded.

### Data extraction and quality assessment

After collecting the findings from all databases, the articles were exported to Microsoft Excel spreadsheet. Newcastle-Ottawa Quality Assessment Scale (NOS) for cross-sectional was used to assess the methodological quality of a study and to determine the extent to which a study has addressed the possibility of bias in its design, conduct and analysis [15]. All the included articles scored (NOS) 7 and more can be considered as “good” studies with low risk.

### Statistical analysis

As the test statistic showed significant heterogeneity among studies (I^2^ = 99.4%, *p* < 0.05) the Random-effects model was used to estimate the DerSimonian and Laird’s pooled effect [16]. Cochran’s Q chi-square statistics and I^2^ statistical test was conducted to assess the random variations between primary studies [17]. In this study, heterogeneity was interpreted as an I^2^ value of 25% = low, 50% = moderate, and 75% = high [18]. In case of high heterogeneity, subgroup analysis and sensitivity analyses were run to identify possible moderators of this heterogeneity. Potential publication bias was assessed by visually inspecting funnel plots and objectively using the Egger’s test (i.e. *p* < 0.05) [19]. To account for any publication bias, we used the trim-and-fill method, based on the assumption that the effect sizes of all the studies are normally distributed around the center of a funnel plot. The meta-analysis was performed using the Stata version 11.0 (Stata Corporation, College Station, Texas, USA) software. Finally, for all analyses, *P* < 0.05 was considered statistically significant.

## Results

### Study selection and data extraction

The search strategy identified 80 articles from PubMed, 60 articles from Google Scholar, 45 articles from Cochrane Library, 10 articles from African Journals Online, 7 articles from Ethiopian’s University online library, and 5 articles by manual search. Of which, 134 were excluded due to duplication, 35 through review of titles and abstracts. Additionally, 31 full-text articles were excluded for not reporting the outcome variable and other reasons. Finally, 11 were included to the prevalence and/ or associated factor analysis on dual contraception use (Fig.1).

**Fig. 1:** Flow chart of study selection for systematic review and meta-analysis of dual contraception use in Ethiopia

### Study characteristics

Different factors such as having open partner discussion, provision of post-test counseling, disclosed HIV status to sexual partner, partner involvement in post-test counseling, and currently on highly active antiretroviral therapy (HAART) were included in this study. Eleven cross-sectional studies with a total of 4080 women living with HIV were included in this review. Regarding the study area, included studies were from SNNPR (south nation nationalities and people representative), Tigray, Amhara, and Oromia (Table 1).

**Table 1:** Descriptive summary of included studies on dual contraceptive method utilization

Author (year of study)	Study area	Sample size	Study region	Prevalence (%)
Mebratu M.et al.(2018) [20]	University of Gondar hospital	376	Amhara	13.2
Solomon W.et al.(2016) [21]	public hospitals of Northern Ethiopia	331	Tigray	23
Markos S.et al.(2019) [22]	Art Clinics in West Zone Health Facilities Oromia, Ethiopia	323	Oromia	25
Dereje B.et al.(2015) [23]	Gebretsadik Shawo Hospital, SNNPR, South West Ethiopia	246	SNNPR	19.8
Meseret W. et al.(2015) [22]	Gondar City, northwest, Ethiopia:	655	Amhara	30
Fewuze A.et al. ABAY(2018) [23]	Tigray Region, Northern Ethiopia	964	Tigray	14.3
Melaku Y.et al.(2014) [3]	Hosanna Hospital, Southern Ethiopia;	403	Amhara	30.9
Addisu P. et al. [24]	ART attendees in health facilities of Gimbie town, West Ethiopia	424	Oromia	30
Yemane B. et al. [25]	HIV Positive Reproductive Age Women in Tigray	364	Tigray	59.9
Assefa A. et al. [26]	HIVPositive Women in Reproductive Age Group, Region, Northwest Ethiopia	409	Amhara	40.9
Alemu T. et al. [27]	HIVPositive Women in Reproductive Age Group, Oromia Region	348	Oromia	85.2

### Prevalence of dual contraceptive use among women living with HIV

A wide-ranging prevalence of dual contraceptive use was observed across different studies included in this review. The overall pooled prevalence of dual contraceptive use among women living with HIV in Ethiopia was 34.08% (95%CI: 20.77–47.38, I^2^ = 99.2%, *p* = < 0.001) (Fig. 2).

**Fig. 2:** Forest Plot for the Prevalence of dual contraception use among women living with HIV in Ethiopia

### Subgroup analysis

Subgroup analysis was employed with the evidence of heterogeneity. In this study, the Cochrane I^2^ statistic was 99.2%, *P* < 0.001, which showed the evidence of marked heterogeneity. Therefore, subgroup analysis was done using the study region and year of study. As a result, dual contraception use among women living with HIV was highest in Oromia region 49.09%, whereas 43.58% in the study conducted between 2015 and 2017 (Figs. 3 and 4).

**Fig. 3:** Subgroup analysis of the pooled prevalence of dual contraception use among women living with HIV based on the study region

**Fig. 4:** Subgroup analysis of the pooled prevalence of dual contraception use among women living with HIV based on year of study

### Publication bias

The funnel plot was assessed for asymmetry distribution of prevalence of dual contraception use among women’s living with HIV by visual inspection (Fig. 5). Egger’s regression test showed a *p*-value of 0.436 with no evidence of publication bias.

**Fig. 5:** Funnel plot with 95% confidence limits of the pooled prevalence of dual contraception use among women living with HIV in Ethiopia

### Sensitivity analysis

This systematic review and meta-analysis showed that the point estimate of its omitted analysis lies within the confidence interval of the combined analysis. Therefore, trim and fill Analysis was no further computed (Fig. 6).

**Fig. 6:** Sensitivity analysis of the pooled prevalence of pooled prevalence of dual contraception use among women living with HIV in Ethiopia

### Determinants of dual contraception use among women living with HIV

The association between having open partner discussion, provision of post test counseling, disclosed HIV status to sexual partner, partner involvement in post-test counseling, and currently on highly active antiretroviral therapy (HAART) with dual contraception use was carried out.

Six studies were included in this category of meta-analysis [3, 20–23] to associate open partner discussion with dual contraception use. Women who discuss openly with sexual partner about dual contraception method were 3.96 times (AOR: 3.96, 95% CI: 2.3–6.8) more likely to use dual contraception as compared to those women who did not have open discussion with sexual partner (Fig. 7).

**Fig. 7:** Forest plot displaying the relationhip between open partner discussion and dual protection use in Ethiopia

Five studies were included in this category of meta-analysis [3, 20–23]. The odds of using dual protection among women living with HIV who counseled during post-test was 4.38 times (AOR: 4.38, 95% CI: 2.93–6.54) more compared with their counterparts (Fig. 8).

**Fig. 8:** Forest plot displaying the association between provision of post-test counseling and dual contraception use in Ethiopia

Four studies were included in this category of meta-analysis [20, 21, 23, 24]. HIV-positive women who disclosed their HIV status to sexual partners were 5.91 times (AOR: 5.91, 95% CI: 4.19–8.33) more likely to use dual contraception as compared to those who did not disclosed their status to sexual partner **(**Fig. 9).

**Fig. 9:** Forest plot displaying the association between disclosed HIV status to sexual partner and dual contraception use in Ethiopia

Tree studies were included in this category of meta-analysis [21–23]. The odd of using dual contraception among women of living with HIV with currently on HAART was 2.92 times (AOR = 2.92, 95% CI: 1.56–5.46) more likely compared with their counterparts (Fig. 10).

**Fig. 10:** Forest plot displaying the association between being on HAART and dual contraception use in Ethiopia

Four studies were included in this category of meta-analysis [3, 20, 23, 24]. The likelihood of using dual contraception among women living with HIV whose partners involved in post test counseling were 3.52 times (AOR = 3.52, 95% CI: 2.3–5.3) more likely to use dual contraception than women whose partners did not involved in post test counseling (Fig. 11).

**Fig. 11:** Forest plot displaying the association between partner involvement in post-test counseling and dual contraception use in Ethiopia

## Discussion

According to the results of this meta-analysis, the pooled prevalence of dual contraception use in Ethiopia was estimated to be 34.08% (95%CI: 20.77–47.38). This finding was lower than the studies done in kenya [28], Tanzania [29], United States of America [30], and systematic review done by Marge Berer [9]. The high dual contraception prevalence in Kenya and Tanzania might be as a result of campaigns to scale-up dual protection use by involving service providers and change in dual-protection counseling. The high use in USA could be due to the high quality and strong integration of Sexual Reproductive Health (SRH) services with services of HIV [31].

Women who ever had open discussion with sexual partner about dual protection were 3.96 times more likely to use dual protection as compared to women who were not. This result is supported by a study conducted Tanzania [32]. This can be explained by the fact that women who openly discuss using dual protection with sexual partner could better understand the importance of dual protection. Additionally, open discussion on using dual protection with sexual partner would give confidence and freedom for both choosing the appropriate contraceptive methods and freedom to negotiate safer sex and birth spacing.

Provision of post-test counseling by health care provider was significant factor to use dual protection among HIV positive women. Those counseled by health care provider to use dual protection after tested positive were 4.3 more odds of using dual contraception. This agrees with a study conducted in Zambia [33], India [34], Tanzania [32], and Kenya [35]. This strongly indicates that counseling of HIV positive women can improve the utilization of dual contraceptive use in preventing sexually transmitted infections and unintended pregnancy. It also indicates that health care providers need to focus on counseling on dual contraception and its benefit to HIV positive women during post-test counseling and during follow up at the ART clinic.

Disclosing HIV status to sexual partners showed statistically significant association with dual contraceptive use among women living with HIV. Women who disclosed HIV status to sexual partner were nearly 5.9 times more likely to utilize dual contraception as compared to those women who did not disclose their status to sexual partners. Similar study findings were observed in different countries: Kenya [36], India [37], and Zambia [33]. It could be due to the fact that disclosure likely facilitates open discussion between partners in relation to HIV infection, dual contraception, and both parties might understand the importance of consistent dual contraceptive use. Moreover, women who disclose their status to their sexual partner might be supported each other and promote to visit health care facilities for counseling which in turn promote dual contraceptive use.

The odds of dual contraceptive use among women with partner’s involvement in post-test counseling were about 3.52 times higher than their counterparts. The finding of this study is consistent with the study done in India [34]. This possible reason might be testing and counseling sexual partners together encourages them to have open discussion while choosing the appropriate contraceptive methods they use.

This review also showed that being currently on highly active antiretroviral therapy (HAART) was significantly associated with dual protection use among women living with HIV. Women who were on (HAART) were nearly 3 times more likely to use dual contraception as compared to their counter parts. This result is supported by study done in Brzail [38]. The possible reason might be being on HAART requires frequent visits to healthcare facilities which may be linked to greater exposure to safe sex counseling, dual protection, greater access to condoms, and health care seeking behavior. Moreover, women who care for themselves by adhering to HAART regimens may have greater odds of also protecting their sexual partners by using condoms consistently.

### Limitations

This meta-analysis was included only articles conducted in the English language, which may have restricted some papers conducted in local language from being included. Additionally, all the included articles were cross-sectional; as a result, the outcome variables might be affected by confounding variables and it might be difficult to address the temporal cause and effect relationship via cross-sectional studies.

## Conclusion

The pooled prevalence of dual contraceptive was low among women living HIV was low in Ethiopia. Having open partner discussion, provision of post-test counseling, disclosed HIV status to sexual partner, partner involvement in post-test counseling, and currently on highly active antiretroviral therapy (HAART were the determinants factors of dual contraceptive in Ethiopia. Therefore, efforts might be made to improve the use of dual contraception by providing simultaneous HIV testing and counseling of women with their partner, promoting open partner discussion, and provision of counseling by health care providers during post testing, and follow up at the ART clinics regarding dual contraception shall be encouraged.

## Data Availability

The data sets generated during the current study are available from corresponding author on reasonable request.

## Abbreviations

AIDS: Acquired immune deficiency syndrome
AOR: Adjusted Odds Ratio
ART: Antiretroviral therapy
CI: Confidence Interval
HAART: Highly active antiretroviral therapy
HIV: Human immune deficiency virus
JBI: Joanna Briggs Institute
MTCT: Mother to child transmission
OR: Odds Ratio
PMTCT: Prevention of mother to child transmission
PRISMA: Preferred Reporting Items for Systematic Review and Meta-Analysis statement
SPSS: Statistical Package for Social Sciences
STI: Sexually transmitted infection
SNNPR: Southern Nation Nationality and Peoples Region
